The article "A comparison of the safety and efficacy of tapinarof and roflumilast topical therapies in the management of mild‐to‐moderate plaque psoriasis" was published in 2024. Journal: Skin Res Technol.

# A comparison of the safety and efficacy of tapinarof and roflumilast topical therapies in the management of mild‐to‐moderate plaque psoriasis

**DOI:** 10.1111/srt.70041

**Published:** 2024-08-29

**Authors:** Hira Ghani, Alicia Podwojniak, Isabella J. Tan, Aarushi K. Parikh, Bianca Sanabria, Babar Rao

**Affiliations:** ^1^ Dermatology Clinical Trials Unit Northwestern University Feinberg School of Medicine Chicago Illinois USA; ^2^ Rowan‐Virtua School of Osteopathic Medicine Stratford New Jersey USA; ^3^ Rutgers Robert Wood Johnson Medical School New Brunswick New Jersey USA

**Keywords:** adverse effects, efficacy, GSK2894512, plaque psoriasis, psoriasis, roflumilast, tapinarof, topical therapy

## Abstract

**Introduction:**

Psoriasis is an immune‐mediated inflammatory skin disease. First‐line topical treatments include steroids, calcineurin inhibitors, vitamin D analogs, and anthralin. Recently, novel topical therapeutics like tapinarof and roflumilast have emerged with unique anti‐inflammatory mechanisms and promising efficacy profiles.

**Materials and methods:**

This review utilized PubMed, SCOPUS, and Web of Science databases to identify recent studies on tapinarof and roflumilast. Criteria focused on efficacy, safety profiles, and therapeutic roles in psoriasis treatment.

**Results:**

Four primary literature articles were identified for tapinarof and five for roflumilast. Both drugs demonstrated strong efficacy with minimal adverse events in treating mild‐to‐moderate plaque psoriasis. Tapinarof showed more frequent but mild adverse effects, while roflumilast had less frequent but more severe side effects.

**Discussion:**

Tapinarof and roflumilast offer once‐daily dosing and successful treatment in restricted areas, potentially enhancing patient adherence. Cost remains a limiting factor, necessitating future comparative studies to evaluate the efficacy, safety, and cost‐effectiveness between the two drugs.

**Conclusion:**

Tapinarof and roflumilast present promising topical treatments for psoriasis, showing efficacy and manageable safety profiles. Further research is crucial to fully elucidate their comparative benefits and drawbacks in clinical practice.

## 1 INTRODUCTION

Psoriasis, a chronic inflammatory skin disorder, presents a global health challenge due to its increasing prevalence and impact on quality of life. Despite existing treatment modalities, accessibility, cost, efficacy, and adverse effects remain significant issues.^1^ This review focuses on the limitations of current therapies and explores the potential of tapinarof 1% cream and roflumilast 0.3% cream as emerging treatments. Tapinarof activates the aryl hydrocarbon receptor to limit immune cell expression, while roflumilast inhibits phosphodiesterase‐4, targeting inflammatory pathways implicated in psoriasis (Figure 1).^2^, ^3^ The Food and Drug Administration (FDA) has approved topical roflumilast for plaque psoriasis treatment in patients aged 12 and older.^4^ The review aims to assess and compare the efficacy and safety of these treatments to guide clinicians and researchers in selecting optimal management strategies for mild‐to‐moderate plaque psoriasis.

The article "A comparison of the safety and efficacy of tapinarof and roflumilast topical therapies in the management of mild‐to‐moderate plaque psoriasis" was published in 2024. Journal: Skin Res Technol.

**FIGURE 1:** Tapinarof and Roflumilast mechanism of action. Left: Tapinarof binds to and activates aryl hydrocarbon receptor (AhR), a ligand‐dependent transcription factor, in the cytoplasm. The now‐activated AhR‐tapinarof complex heterodimerizes with the AhR nuclear translocator (ARNT). The AhR‐tapinarof/ARNT complex induces gene expression that leads to the downregulation of proinflammatory cytokines, including interleukin (IL) 17, which is involved in the pathogenesis of psoriasis. Right: Roflumilast inhibits the phosphodiesterase‐4 (PDE‐4) isoenzyme, consequently increasing intracellular concentrations of the secondary messenger cyclic adenosine monophosphate (cAMP) in affected cells. This suppresses inflammation through a decreased release of inflammatory cytokines.

## 2 MATERIALS AND METHODS

We conducted a literature review utilizing Pubmed, SCOPUS, and Web of Science databases to gather recent articles focusing on tapinarof and roflumilast for psoriasis treatment. Using the NLM Medical Subject Heading (MeSH) to derive search terms, we constructed strings including (“tapinarof” OR “roflumilast”) AND (“psoriasis”) AND (“adverse effects”) AND (“efficacy”).

Inclusion criteria were defined as articles involving primary data (e.g., randomized controlled trials, cohort studies, retrospective studies, case studies, case series), human subjects only, published from 2018 to 2023, and addressing the efficacy and safety profile of either roflumilast or tapinarof for plaque psoriasis treatment. Priority was given to primary sources, with secondary sources considered to supplement missing information. Exclusion criteria included abstracts, articles lacking full text, studies in progress, and those focusing on treatment options other than tapinarof or roflumilast for psoriasis.

Two reviewers (A.P. and H.G.) performed full‐text appraisal, assessing relevance, proper data reporting, and clinical outcomes. The review process adhered strictly to the defined criteria, ensuring the inclusion of relevant and accurate studies. Additional pertinent articles were included if identified beyond the original search terms. A detailed summary of the study selection process is provided in Figure 2.

The article "A comparison of the safety and efficacy of tapinarof and roflumilast topical therapies in the management of mild‐to‐moderate plaque psoriasis" was published in 2024. Journal: Skin Res Technol.

**FIGURE 2:** Study selection process.

## 3 RESULTS AND DISCUSSION

### 3.1 Tapinarof efficacy

Robbins et al. report the findings of a phase 2 clinical trial on the efficacy of the application of 0.5% and 1% tapinarof cream once or twice daily therapy for adults with plaque psoriasis (Table 1). This randomized, double‐blind multicenter study included 175 participants who completed a 12‐week treatment. In the study, treatment success was measured by the Physician Global Assessment (PGA) score of 0 or 1, and additional outcomes included >75% improvement in Psoriasis Area and Severity Index (PASI). Tapinarof was found to statistically improve psoriasis lesions in both concentration groups and duration groups as measured by PGA and PASI (*p* < 0.001, *p* < 0.05).^5^ Improvement measured by PGA was maintained for 4 weeks post‐treatment. Clinical improvements were noted approximately 2 weeks post‐treatment initiation.^5^

**TABLE 1:** Summary of primary studies included in this review.

Authors	*N* =	Duration of treatment	Efficacy	Adverse effects
**Tapinarof**				
Robbins et al. (NCT02564042)	175	12 weeks	Significant improvement in both PGA and PASI (*p* < 0.001, *p* < 0.05); improvement (PGA) sustained for 4 weeks post‐treatment.	Total TEAEs in 46% of participants (mild‐moderate). Folliculitis (9%). Contact dermatitis. (8%). Additional effects: application site dermatitis, irritation, allergic dermatitis, decreased monocytes, headache (1% each).
Stein‐Gold et al. (NCT02564042)	175 (same trial as above)	12 weeks (same trial as above)	The same outcomes as above; also included PSD scores in tapinarof cohort were significantly reduced compared to vehicle (*p* < 0.05).	As above.
Lebwohl/Stein et al. (NCT03956355, NCT03983980)	Psoaring 1: 510 Psoaring 2: 512	12 weeks	Primary endpoint of PGA score (0 or 1), achieved with significance with tapinarof use in both trials 1 and 2 (*p* < 0.001). Secondary endpoints of PASI 75 and PASI 90 were achieved with significance with tapinarof use (*p* < 0.001).	PSOARING 1: Treatment‐related adverse effects reported: 171 (50.3%). Folliculitis: 80 (23.5%) Contact dermatitis: 17 (5.0%). Nasopharyngitis: 25 (7.4%) Additional effects: Upper respiratory infection, pruritus, headache.
				PSOARING 2: Treatment‐related adverse effects reported: 187 (54.5%). Folliculitis: 61 (17.8 %). Contact dermatitis: 20 (5.8%). Nasopharyngitis:14 (4.1%). Additional effects: Upper respiratory infection, pruritus, headache.
Strober et al. (NCT04053387)	PSOARING III: 763	40 additional weeks (52 total)	40.9% of participants achieved a complete disease clearance, measured as PGA of 0. 85.8% of patients reported subjective satisfaction.	Treatment‐related adverse effects reported: 210 (27.5%). Folliculitis: 173 (22.7%). Contact dermatitis: 42 (5.5%). Upper Respiratory infection: 36 (4.7%). Additional effects: nasopharyngitis, pruritus, acne, back pain.
Roflumilast				
Lebwohl/Kirckik et al. (NCT04311363, NCT04211389) Nicholas et al.	DERMIS‐1: *n* = 439 DERMIS‐2: *n* = 442	8 weeks	Roflumilast cohort demonstrated a statistically significant increase in IGA. DERMIS 1: 42.4% (*p* < 0.001) DERMIS 2: 37.5% (*p* < 0.001). Significant improvement in 8/9, and 9/9 of secondary outcomes in DERMIS 1,2, respectively.	Total TEAEs. DERMIS 1: (25.2%) with roflumilast vs. (23.5%) with placebo. DERMIS 2: (25.9%) with roflumilast vs. (18.4%) with placebo. Most common: urticaria at the application site experienced by 0.3% of participants. Additional adverse effects (DERMIS 1): diarrhea (3.1%), headaches (2.4%), and insomnia (1.4%).
Lebwohl/Papp et al. (NCT03638258)	331	12 weeks	Outcome of a clear or almost clear IGA score at week 6 was observed in 28% of the patients in the roflumilast 0.3% group, 23% in the roflumilast 0.15% group, and 8% in the placebo group (*p* < 0.001).	Frequency of ADE (6% for roflumilast 0.3%) (3% for roflumilast 0.15%), (7% for vehicle). Most common ADEs: nasopharyngitis and URI symptoms. Nausea and diarrhea were seen in (>1%).
Draelos et al. (NCT03638258)	331	12 weeks	Post hoc analysis of Lebwohl/Papp. At week 6, IGA of 0 to 1 met (roflumilast 0.3%, 27.2%; roflumilast 0.15%, 22.3%; vehicle, 6.3%; (nominal *p* ≤ 0.026). IGA of 0 to 1 plus a two‐grade improvement for Roflumilast (0.3%) at weeks 6, 8, and 12 and in those treated with roflumilast 0.15% at weeks 8 and 12 (nominal *p* < 0.05).	Reports of application‐site pain lower in roflumilast patients vs. vehicle (1.8−2.1% vs. 3.6%). Reports of ‘no sensation’, ‘slight warm, tingling sensation; not really bothersome’ on post‐baseline assessments. Roflumilast (≥ 97.0%) vehicle and (≥ 96.2%).
Papp et al. (NCT03392168)	97	4 weeks	Both 0.5% or 0.15% roflumilast doses showed improvement in TPSS; for roflumilast 0.5% (*p* = 0.0007) and 0.15% (*p* = 0.0011).	TEAEs were limited to the application site, with no differences between drug and vehicle; application site erythema and pain, nasopharyngitis, and muscle strain were reported. No patient discontinuation due to ADEs.

Stein‐Gold et al. reported additional outcomes of the same study, including Psoriasis Symptom Diary (PSD) scores and the patients’ impressions of symptom severity and pruritus.^6^ The PSD tool is a validated, self‐reported tool specific for psoriasis and uses 16 ± 6 questions to assess subjective measures of psoriasis symptoms.^7^ The PSD scores in the tapinarof‐treated cohort were significantly reduced compared to the vehicle control (*p* < 0.05).^6^ Patient‐reported severity scores and subjective measures of pruritis were also significantly improved in all tapinarof‐treated groups compared to vehicle controls (*p* < 0.05).^6^

The article "A comparison of the safety and efficacy of tapinarof and roflumilast topical therapies in the management of mild‐to‐moderate plaque psoriasis" was published in 2024. Journal: Skin Res Technol.

Lebwohl et al., report the findings of the PSOARING 1 and PSOARING 2 Trials, two identical phase III trials in which 510 (340 tapinarof, 170 vehicle) and 512 (343 tapinarof, 172 vehicle) patients were enrolled, respectively.^8^ The primary endpoint of the PGA score (0 or 1), was achieved with statistical significance in both trials, 1 and 2, (*p* < 0.001). Secondary endpoints of PASI 75 and PASI 90 also reached significance in treatment groups of both trials, as compared to vehicle controls (*p* < 0.001). Such results are similar to the existing phase II trials.^5^

Results from PSOARING 3, the phase III trial includes 1‐year safety and efficacy of tapinarof for plaque psoriasis are reported in Strober et al. In this trial, patients had to have completed 12 weeks with tapinarof or the vehicle as described in aforementioned trials, PSOARING 1 and 2.^9^ These patients, of which 763 participated, were eligible for an additional 40 weeks of treatment, totaling 52 weeks. This trial showed that 1% concentration cream had continued improvement beyond 12 weeks and was well tolerated up to 52 weeks. Overall, 40.9% of participants achieved a complete disease clearance, measured as PGA of 0.^9^ Remission was achieved for an average of 4 months for patients who had achieved PGA of 0 during any time point in the trial. Further, regarding patient‐reported satisfaction, 85.8% reported satisfaction with the ease of managing their psoriasis with tapinarof, and 62.9% of patients indicated agreeing that the drug cleared their lesions and prevented recurrence.^10^

### 3.2 Tapinarof safety profile

Phase 2 trials did not identify statistically significant adverse effects stemming from tapinarof use, as measured by both investigator‐reported and patient‐reported tolerability scores.^6^ 46% of patients experienced mild‐moderate adverse effects, and 68% came from the 1% twice‐daily cohort. Folliculitis, contact dermatitis, and other application site dermatitis were the most commonly reported. Contact dermatitis was the most common reason for treatment discontinuation, seen in 3% of participants.^5^ The safety profile and tolerability of tapinarof are well documented in the PSOARING trials. PSOARING 1 and 2 identified no significant differences between the treatment and vehicle cohorts regarding laboratory values, vitals, physical exam findings, or electrocardiogram measures.^8^ Just over half of the participants in each trial (50.3% and 54.5%, respectively) reported adverse effects, with the most commonly reported being folliculitis (23.5%, 17.8%, respectively) and contact dermatitis (5.0% and 5.8%, respectively). Of these, folliculitis severity led to discontinuation (1.8% and 0.9%), and contact dermatitis led to discontinuation (1.5% and 2.0%).^8^ Additional reported findings included headache (3.8% in both trials).^8^ The incidence of patient‐reported burning, stinging, or pruritus was low. The most commonly reported adverse events following prolonged use of tapinarof were noted to be similar to short‐term use. In the PSOARING 3 trials, 27.5% of participants reported adverse effects, the most common being folliculitis and contact dermatitis. Of these, discontinued use was reported in 1.2% and 1.4% of patients secondary to folliculitis and contact dermatitis, respectively.^9^

The article "A comparison of the safety and efficacy of tapinarof and roflumilast topical therapies in the management of mild‐to‐moderate plaque psoriasis" was published in 2024. Journal: Skin Res Technol.

### 3.3 Roflumilast efficacy

Lebwohl and Kircik et al. postulated the superior efficacy of roflumilast 0.3% cream compared to the placebo in the treatment of chronic plaque psoriasis based on the results from two phase 3, randomized, double‐blind, controlled, multicenter trials (DERMIS‐1 [trial 1; *n* = 439] and DERMIS‐2 [trial 2; *n* = 442]). Patients with ages 12 years and older with 2% to 20% of body surface area consisting of plaque psoriasis were randomized in a 2:1 ratio to receive roflumilast cream, 0.3% (trial 1: *n* = 286; trial 2: *n* = 290), or vehicle cream (trial 1: *n* = 153; trial 2: *n* = 152) once daily for 8 weeks. The primary endpoint was the Investigator Global Assessment (IGA) score improvement from the baseline (score range, 0–4) at week 8, along with 9 secondary outcomes, including intertriginous IGA success, 75% reduction in PASI score, and Worst Itch Numeric Rating Scale score of 4 or higher at baseline achieving a 4‐point reduction (WI‐NRS success) at week 8. The Roflumilast cohort demonstrated a statistically significant increase in IGA success percentages at week 8 than the vehicle cohort (trial 1: 42.4% vs. 6.1% [95% CI, 32.3%−46.9%]; trial 2: 37.5% vs. 6.9% [95% CI, 20.8%−36.9%]; *p* < 0.001 for both). Statistically significant differences favoring roflumilast over placebo were observed for 8 out of 9 secondary endpoints in trial 1, and all 9 secondary endpoints in trial 2, demonstrating the superior efficacy of roflumilast.^11^

Results from a double‐blind, phase 2b study by Lebwohl and Papp et al. where adults with plaque psoriasis were randomly assigned to use roflumilast 0.3% cream, roflumilast 0.15% cream, or placebo once daily for 12 weeks also concluded the potency of roflumilast cream in the treatment of psoriasis.^12^ The primary outcome of a clear or almost clear IGA score at week 6 was observed in 28% of the patients in the roflumilast 0.3% group, in 23% in the roflumilast 0.15% group, and 8% in the placebo group (*p* < 0.001).^12^ The mean baseline PASI scores (a secondary outcome measure) were 7.7 in the roflumilast 0.3% group, 8.0 in the roflumilast 0.15% group, and 7.6 in the vehicle group (range, 0 to 72, with higher scores indicating worse disease).^12^ Nicolas et al. also summarize roflumilast efficacy and safety in the DERMIS‐1 and DERMIS‐2 clinical trials. The IGA success rate of 42.4% with roflumilast 0.3% cream compared to 6.1% with the vehicle in DERMIS‐1 (32.3%−46.9%; *p* < 0.001), and the IGA success rate of 37.5% with roflumilast 0.3% cream compared to 6.9% with the vehicle in DERMIS‐2 (20.8%−36.9%; *p* < 0.001) indicates the statistically significant efficacy of roflumilast.^4^ Overall, topical roflumilast cream has shown to be effective in treating sensitive, intertriginous areas, and may be a good alternative to existing systemic therapy with far more notable adverse events.^4^

The article "A comparison of the safety and efficacy of tapinarof and roflumilast topical therapies in the management of mild‐to‐moderate plaque psoriasis" was published in 2024. Journal: Skin Res Technol.

Papp et al. assessed the safety and efficacy of roflumilast in a phase 1/2a study comprising a single‐dose, open‐label cohort of 0.5% roflumilast cream applied to 25 cm^2^ psoriatic plaques (cohort 1), and a 28‐day, double‐blinded cohort with 1:1:1 randomization to 0.5% or 0.15% roflumilast cream, or the vehicle (cohort 2).^13^ The primary efficacy endpoint was met for both 0.5% or 0.15% roflumilast cream doses as demonstrated by Target Plaque Severity Score [TPSS] × Target Plaque Area [TPA]) improvement at week 4, which was statistically significant for roflumilast 0.5% (*p* = 0.0007) and 0.15% (*p* = 0.0011) versus the placebo. For both roflumilast doses, 66%−67% improvement from the baseline was observed at week 4, as opposed to 38% improvement for the vehicle. A post‐hoc analysis of the aforementioned phase 2b clinical trial to evaluate the tolerability and efficacy of roflumilast cream when applied daily for 331 patients, of which 160 (48%) had psoriasis involving the face and/or intertriginous areas.^13^ At week 6, an IGA of 0 to 1 was met by patients receiving roflumilast (roflumilast 0.3%, 27.2%; roflumilast 0.15%, 22.3%; vehicle, 6.3%; nominal *P* ≤ 0.026). The percentage of patients with an IGA of 0 to 1 plus a two‐grade improvement was also higher for the patients treated with roflumilast 0.3% at weeks 6, 8, and 12 and in those treated with roflumilast 0.15% at weeks 8 and 12 (nominal *p* < 0.05).^14^ Overall, it can be concluded that once‐daily application of roflumilast cream is associated with a high efficacy and tolerability profile at both 0.5% and 0.15% doses when compared to existing topical therapies for chronic plaque psoriasis.

The article "A comparison of the safety and efficacy of tapinarof and roflumilast topical therapies in the management of mild‐to‐moderate plaque psoriasis" was published in 2024. Journal: Skin Res Technol.

### 3.4 Roflumilast safety profile

Roflumilast exhibits tolerability and safety with minimal risk of adverse events. The incidence of treatment‐emergent adverse events (TEAE) in the DERMIS trials was 25.2% with roflumilast in contrast to 23.5% with placebo in trial 1, and 25.9% with roflumilast when compared to 18.4% with placebo in trial 2.^11^ The incidence of serious adverse events (SAE) was the same with roflumilast and vehicle in trial 1, and 0% with roflumilast versus 0.7% with the vehicle in trial 2.^11^ Approximately 1% of patients discontinued treatment with roflumilast due to adverse reactions compared with 1.3% treated with the placebo. The most common TAE seen with roflumilast was urticaria at the application site experienced by 0.3% of participants.^4^ In a phase 2 study by Gooderham et al., TEAE occurred in 2 (2.2%) patients receiving roflumilast, including mild rash and moderate application site pain, and only 1 (1.1%) patient discontinued the study due to a drug‐related AE.^15^ Additional reported adverse effects included diarrhea (3.1%), headaches (2.4%), and insomnia (1.4%) in DERMIS 1,^16^, ^17^ and application site erythema and pain, nasopharyngitis, and muscle strain were additionally reported.^13^, ^17^, ^18^

### 3.5 Clinical relevance

Existing topical treatments for psoriasis (steroids, vitamin D derivatives, TCIs) are limited by adverse effects. Tapinarof and roflumilast offer non‐steroidal options, preferred by patients for ease of use. Tapinarof allows chronic use with limited site restrictions,^19^ and showing 4‐month efficacy.^20^ Roflumilast is effective in intertriginous areas, with once‐daily dosing.^16^ Tapinarof lacks data on combination therapy and specific patient populations. Both drugs are costly, with tapinarof at $1405^20^ and roflumilast at $825^16^, posing challenges in adherence. Roflumilast lacks data on hepatic disease.^16^ Direct comparator studies between tapinarof and roflumilast are needed to ascertain the clinical outcomes, safety, and efficacy of one over the other.

## 4 CONCLUSION

Both tapinarof 1% cream and roflumilast 0.3% cream effectively treat mild‐to‐moderate plaque psoriasis with minimal adverse events, improving compliance with their water‐based formulations. Tapinarof has more frequent but less severe side effects compared to roflumilast. However, their high cost and prior authorization requirements limit accessibility. Further research, especially in pediatric populations, is necessary to evaluate long‐term efficacy and tolerability.

## CONFLICT OF INTEREST STATEMENT

The authors declare no conflicts of interest.

## ETHICS STATEMENT

Not applicable.

The article "A comparison of the safety and efficacy of tapinarof and roflumilast topical therapies in the management of mild‐to‐moderate plaque psoriasis" was published in 2024. Journal: Skin Res Technol.

## PATIENT CONSENT STATEMENT

Not applicable.

## Data Availability

The data that supports the findings of this review are available from publicly accessible sources and repositories. All references and citations to the primary studies, datasets, and literature sources utilized in this review are listed in the reference section.
